RETRACTED

# Catestatin Increases the Expression of Anti-Apoptotic and Pro-Angiogenetic Factors in the Post-Ischemic Hypertrophied Heart of SHR

**DOI:** 10.1371/journal.pone.0102536

**Published:** 2014-08-06

**Authors:** Claudia Penna, Teresa Pasqua, Daniela Amelio, Maria-Giulia Perrelli, Carmelina Angotti, Francesca Tullio, Sushil K. Mahata, Bruno Tota, Pasquale Pagliaro, Maria C. Cerra, Tommaso Angelone

**Affiliations:** 1 Department of Clinical and Biological Sciences, University of Turin, Torino, Italy; 2 Department of Biology, Ecology and Earth Sciences, University of Calabria, Arcavacata di Rende, Italy; 3 VA San Diego Healthcare System, University of California, San Diego, California, United States of America; 4 National Institute of Cardiovascular Research, Bologna, Italy; University-Hospital of Parma, Italy

## Abstract

**Background:**

In the presence of comorbidities the effectiveness of many cardioprotective strategies is blunted. The goal of this study was to assess in a hypertensive rat model if the early reperfusion with anti-hypertensive and pro-angiogenic Chromogranin A-derived peptide, Catestatin (CST:hCgA_352–372_; CST-Post), protects the heart *via* Reperfusion-Injury-Salvage-Kinases (RISK)-pathway activation, limiting infarct-size and apoptosis, and promoting angiogenetic factors (*e.g.,* hypoxia inducible factor, HIF-1α, and endothelial nitric oxide synthase, eNOS, expression).

**Methods and Results:**

The effects of CST-Post on infarct-size, apoptosis and pro-angiogenetic factors were studied in isolated hearts of spontaneously hypertensive rats (SHR), which underwent the following protocols: (a) 30-min ischemia and 120-min reperfusion (I/R); (b) 30-min ischemia and 20-min reperfusion (I/R-short), both with and without CST-Post (75 nM for 20-min at the beginning of reperfusion). In unprotected Wistar-Kyoto hearts, used as normal counterpart, infarct-size resulted smaller than in SHR. CST-Post reduced significantly infarct-size and improved post-ischemic cardiac function in both strains. After 20-min reperfusion, CST-Post induced S-nitrosylation of calcium channels and phosphorylation of RISK-pathway in WKY and SHR hearts. Yet specific inhibitors of the RISK pathway blocked the CST-Post protective effects against infarct in the 120-min reperfusion groups. Moreover, apoptosis (evaluated by TUNEL, ARC and cleaved caspase) was reduced by CST-Post. Importantly, CST-Post increased expression of pro-angiogenetic factors (*i.e.,* HIF-1α and eNOS expression) after two-hour reperfusion.

**Conclusions:**

CST-Post limits reperfusion damages and reverses the hypertension-induced increase of I/R susceptibility. Moreover, CST-Post triggers antiapoptotic and pro-angiogenetic factors suggesting that CST-Post can be used as an anti-maladaptive remodeling treatment.

RETRACTED

## Introduction

The presence of comorbidities including hypertension and myocardial hypertrophy has been reported to blunt the efficacy of cardioprotective protocols such as ischemic postconditioning (I-PostC) and to alter expression and responsiveness of several kinases, including those involved in the so-called *Reperfusion-Injury-Salvage-Kinases* (RISK)-pathway [1]–[4] ^.^ Although (RISK)-pathway activation by I-PostC plays a causal role in cardioprotection in normal rodents, I-PostC effectiveness is compromised in the hypertrophied hearts of spontaneously hypertensive rats (SHR) [1], [5], [6]. Therefore there is a compelling need to find cardioprotective strategies (*e.g.* pharmacological-PostC, P-PostC) [2], [7] for subjects affected by comorbidities.

Catestatin (CST:hCgA_352–372_), a 21-amino-acid derivate of chromogranin A (CgA) [8]–[12] displays hypotensive/vasodilatory properties and counteracts excessive systemic and/or intra-cardiac excitatory stimuli (*e.g*., catecholamines and endothelin-1) [9]–[10]. Produced also by the myocardium [12], CST affects heart performance by modulating inotropy, lusitropy and coronary tone through a NO-dependent mechanism [8]–[10], [13]. Notably, hypertensive patients have lower CST levels than their normotensive counterparts [11]. In fact, CST restores normal blood pressure in CgA knockout mice, which represents monogenic-model of mouse hypertension [11] CST also promotes angiogenesis/arteriogenesis and vasculogenesis in the unilateral mouse hind limb ischemia model [14]. Recently it has been shown that CST activates a PI3K/Akt/NOS-dependent pathway [8]–[10] and elicits cardioprotection in healthy rodent hearts [15], [16]. Importantly, this CST-recruited anti-apoptotic PI3K/Akt/NOS dependent pathway appears to elicit its PostC cardioprotective effects through a mechanism, which also involves mitochondrial K_ATP_ channels and redox-signaling [15], [16]. Moreover, in non-ischemic hearts, CST induces protein S-nitrosylation (SNO) [13], which is emerging as an important reaction in relation to the cardioprotective redox signaling [17]–[19] This information prompted us to test whether CST can improve post-ischemic myocardial remodeling, in which both anti-apoptotic and pro-angiogenetic processes play critical role [20], [21]. Specifically, we hypothesize that CST, given at the early reperfusion, would trigger cardioprotective pathways, including phosphorylation and SNO of critical cardiac proteins in the cardiac hypertrophic model of SHR. Given the anti-apoptotic and pro-angiogenetic properties of CST in normotensive rats, we also hypothesize that CST would slow-down apoptosis and augment the expression of the early pro-angiogenetic factor, namely hypoxia-inducible factor-1 (HIF-1α) [22], [23] in SHR, *i.e.,* a polygenic-model of rodent hypertension [24] The involvement of HIF-1α is of relevance, due to its central role in preconditioning [22], [23] and its redox sensitive expression [22].

RETRACTED

**Figure 1:** Experimental protocols. Before ischemia, hearts were randomly allocated to 1 of the experimental groups. Sham groups hearts were buffer perfused for a total of 90 or 190-Post was infused during the initial 20 minutes of reperfusion only, inhibitors were infused during the final 5 minutes of stabilization, as indicated by the lines under the bars, and during the initial 20 minutes of reperfusion.

## Methods

### Animals

Ethics Statement: the experiments were conducted in accordance with the Directive 2010/63/EU of the European Parliament and were approved and supervised by the ethics committee of the Department of Pharmacy, Health and Nutritional Sciences, University of Calabria and by the ethics committee of the University of Torino. All surgery was performed under anesthesia and all efforts were made to minimize animal suffering.

Experiments were conducted in age-matched SHR and WKY male rats (450–500 g; 6-month-old; Janvier, St Berthevin Cedex-France). Animals were housed under controlled lighting and temperature conditions with free access to standard rat chow and tap water [24], [25]. Blood pressure (BP) was measured daily by a programmed electro-sphygmomanometer (BP-2000 series II; Blood pressure analysis system. Visitech System) in order to confirm the normotensive/hypertensive conditions of the animals used in this study. BP measured before each experiment by tail-cuff method was: WKY: Systolic BP = 122±3 mmHg and Diastolic BP = 90±2 mmHg; SHR: Systolic BP = 182±4 mmHg and Diastolic BP = 143±2 mmHg.

### Isolated heart perfusion

Rats were anesthetized by i.p. of ethyl carbamate (2 g/kg rat) [8], [13], and hearts were rapidly excised, weighed and transferred in ice-cold Krebs–Henseleit buffer solution (KHS) containing (in millimoles) NaCl 113, KCl 4.7, NaHCO_3_ 25, MgSO_4_ 1.2, CaCl_2_ 1.8, KH_2_PO_4_ 1.2, glucose 11, mannitol 1.1, Na-pyruvate 5 (pH 7.4; 37°C; 95% O_2_/5% CO_2_) [9], [15] for immediate aorta cannulation. Retrograde perfusion was conducted at constant flow-rate with KHS at 37°C. Heart weights were: WKY: 1,75±0,18 g; SHR: 2,25±0,2 g. Therefore the flow was adjusted according to heart weight during stabilization to obtain a perfusion pressure of 80–100 mmHg and kept constant (9±1 ml/min/g) thereafter. To avoid fluid accumulation, the left ventricle (LV) was pierced. A water-filled latex balloon, connected to a pressure transducer (BLPR; WRI, Inc., Saratota, FL), was inserted through the mitral valve into the LV, to allow cardiac mechanical parameters recording. A second pressure transducer located above the aorta recorded coronary pressure (CP). Inotropism was evaluated in terms of left ventricular pressure (LVP; mmHg, index of contractile activity), maximal value of the first LVP derivative [+(LVdP/dT)_max_; in mmHg/sec, index of maximal LV contraction rate] and end diastolic ventricular pressure (EDVP; mmHg, index of contracture) [8], [13], [26]. LVP and CP were recorded throughout the experiment using PowerLab data acquisition system and analyzed using Chart software (ADInstruments, Oxford-UK).

RETRACTED

### Experimental protocol (Fig. 1)

In hearts subjected to I/R protocols ischemia and reperfusion were obtained just stopping and restarting the perfusion pump. In order to analyze the damages and molecular effects induced by the experimental maneuvers, after the 30 min ischemia, hearts were subjected to either a period of 120-min of reperfusion (*Long reperfusion groups*) or a period of 20-min of reperfusion only (*Short reperfusion groups*).

#### Long reperfusion groups

In order to have a reference group for the I/R and CST effects, hearts from normotensive animals (WKY, n = 18) were harvested and allowed to stabilize for 40-min. After the stabilization period, hearts were divided in three groups (WKY_Sham, WKY_I/R and WKY_CST-Post; *Groups 1–3*). In *Group 1* (WKY_Sham, n = 6), hearts underwent additional 150-min perfusion only (total 190-min perfusion). In *Group 2* (n = 6) and *Group 3* (n = 6) hearts were subjected to a specific protocol, which consisted in 30-min of global no-flow ischemia and a period of 120-min of reperfusion. In the WKY_CST-Post (*Group 3*), CST (75 nM) was infused for 20-min at the beginning of 120-min reperfusion [15], [16].

After the stabilization period, hearts from hypertensive animals were subjected to the same protocols. In particular, in *Group 4* (SHR_Sham, n = 6), SHR hearts underwent 190-min perfusion only. In *Group 5* (SHR_I/R, n = 6), hearts were exposed to 30 min ischemia and then to 120-min reperfusion. In *Group 6* (SHR_CST-Post; n = 6), CST (75 nM), was infused for 20-min at the beginning of 120-min reperfusion [15], [16].

In *Groups 7 and 8*, the action of CST-Post was studied in SHR hearts in the presence of specific inhibitors of pivotal kinases in cardioprotection, namely the PKC inhibitor, chelerythrine (CHE, 5 µM; SHR_CST-Post+CHE, Group 7, n = 6) [27], or the PI3K/Akt inhibitor, Wortmannin (WN, 0.1 µM; SHR_CST-Post+WN, Group 8, n = 6) [28]. The inhibitors were infused 5-min before and 20-min after ischemia [16], [28]. The inhibitors alone at these concentrations do not affect I/R damages [27]–[30].

RETRACTED

#### Short reperfusion groups

In *Group 9*, (WKY_Sham-short, n = 6) SHR hearts underwent 90 min perfusion only. In *Group 10*, WKY hearts (WKY_I/R-short, n = 6) were exposed to 30-min ischemia and then to 20-min reperfusion only. In *Group 11* (WKY_CST-Post-short, n = 6), hearts were perfused with CST (75 nM) during the 20-min of reperfusion [15], [16].

In *Groups 12–14* (SHR_Sham-short, n = 6; SHR_I/R-short, n = 6; SHR_CST-Post-short, n = 6), SHR hearts underwent protocols similar to those of Groups 9–11.

### Assessment at 120-min reperfusion

#### Infarct size

Infarct areas were assessed at the end of the 120-min reperfusion as previously described [5], [15]–[17], [26]–[28] and the necrotic mass was expressed as a percentage of total left ventricular mass which was considered as risk area. Briefly, at the end of reperfusion, each heart was removed from perfusion apparatus, and the left ventricle (LV) was dissected into 2–3 mm circumferential slices. Following 20-min of incubation at 37°C in 0.1% solution of nitro-blue-tetrazolium in phosphate buffer, unstained necrotic tissue was carefully separated from stained viable tissue by an independent observer. The weights of necrotic and non-necrotic tissues were determined and the necrotic mass was expressed as a percentage of risk area [5], [15]–[17], [26]–[28].

#### Apoptosis

Since in *hypertrophic hearts* apoptotic remodeling is particularly important [31], we studied the level of apoptosis in SHR hearts subjected to 30-ischemia and 120-min reperfusion with and without CST, respectively. TUNEL staining was performed according to the manufacturer (in situ Cell Death Detection Kit, POD from Roche Diagnostics-Germany) [32]. Sections were rehydrated and incubated with proteinase K (20 µg/mL) at 37°C for 20-min. They were washed twice with PBS, and endogenous peroxidase was quenched with 0.3% H_2_O_2_ in PBS for 15-min. Slides were then rinsed and incubated with TUNEL in a humidified box (37°C, 60-min); the reaction was blocked by 3% BSA in PBS at room temperature. Horseradish peroxidase (HRP)-conjugated antibodies were added and incubated at 37°C. Negative controls were obtained by using the same protocol without terminal deoxynucleotidyl transferase (TdT) enzyme (Fig. 2 panel H). Nuclei were counterstained with hematoxylin. Apoptotic Index (AI) was calculated as 100×(number of TUNEL-positive myocyte nuclei per field/total number of myocyte nuclei per field). For each condition, four randomly selected fields were evaluated and averaged [32].

RETRACTED

**Figure 2:** I/R Injury (infarct size and apoptosis) after 30-min ischemia and 120-min reperfusion. Infarct size (IS): the amount of necrotic tissue is expressed as percentage of the left ventricle (% IS/LV), which is considered the risk area. Panel A: effects of CST-Post in normotensive (WKY) or hypertensive (SHR) hearts. Panel B: effects of CST-Post in hypertensive (SHR) heart in the presence of antagonists. TUNEL analysis: the apoptotic index of the cardiac muscle is in panel C. Tunel positive cardiomyocyte nuclei are shown by red arrows in panel D (WKY_Sham), panel E (SHR_Sham), panel F (SHR_I/R), and panel G (SHR_CST-Post). Negative control (panel H) is obtained by using the same protocol without TdT enzyme. Immunohistochemical localization of connexin 43 (green arrows) in the ventricular sections of SHR_Sham (panel I), SHR_I/R (panel L), and SHR_CST-Post (panel M). **p<0.01, *p<0.05. Two way ANOVA, (n = 6 for each group).

Since cleaved caspase 3 and apoptosis repressor with caspase recruitment domain (ARC) are highly involved in apoptosis induced by I/R injury [33], the expression and localization of ARC and cleaved caspase 3 was investigated in SHR ventricle of both CST treated and untreated hearts. Cleaved caspase 3 and ARC expression were analyzed by Western blotting (WB) on ventricular homogenates as previously described [27], [28], [34]. Ventricular cleaved caspase 3 and ARC localization was immune-histochemically evaluated by using a HRP/DAB detection kit (Abcam, Cambridge, MA-USA). Ventricular sections were deparaffined, rehydrated in PBS and pre-treated with H_2_O_2_ to remove endogenous peroxidase activity, incubated for 1-h with Protein Block, and then overnight with polyclonal rabbit cleaved caspase 3 (1∶1000; Sigma-Aldrich St Louis, MO-USA) and ARC antibodies (1∶100; Santa Cruz Biotechnology) at 4°C. Slides were then washed in PBS and incubated with Biotinylated goat anti-rabbit IgG and subsequently with streptavidine peroxidase complex. The signal was visualized by using diaminobenzidine (DAB) as the final chromogen. Ventricular myocytes were discriminated by polyclonal connexin 43 antibody (1∶100; Santa Cruz Biotechnology), by using the above described immunohistochemical protocol.

#### HIF-1α

HIF-1α is involved in long-term cardioprotection and its levels increase within 2-hours of reperfusion [22], [35]. HIF-1α mRNA levels were also evaluated by RT-PCR in 6 additional samples collected after 2-hours reperfusion, for each experimental condition. To evaluate gene expression, at the end of experiments the left ventricles were excised, homogenized with a motor-driven homogenizer and total RNA was isolated using the Trizol reagent (Invitrogen, Milan-Italy), according to the manufacturer’s instructions. RNA integrity was confirmed by visualization of distinct 18S–28S bands after electrophoresis on 1.5% agarose gels stained with ethidium bromide. To remove contaminating genomic DNA, 1 µg of RNA was treated with Rnase free Dnase (RQ1, Promega, Qiagen, Milan-Italy) and then reverse transcribed using Moloney-murine-leukaemia virus reverse transcriptase (MLV-RT; Invitrogen). As negative controls, duplicate RNA samples were incubated in the same buffer with no MLV-RT. Two µl of cDNAs were used for PCR using gene-specific primers. For HIF-1α, the PCR conditions were 1-min at 94°C, 1-min at 56°C, and 1-min at 72°C for 35 cycles using the following primers: forward, 5′-GCTGATTTGTGAACCCATTC-3′ and reverse: 5′-CTGTACTGTCCTGTGGTGAC-3′, generating a 155-bp product. For glyceraldehyde-3-phosphate dehydrogenase, the PCR conditions were 1-min at 94°C, 1-min at 58°C, and 1-min at 72°C for 20 cycles using the following primers: forward, forward: 5′-ACCACAGTCCATGCCATCAC-3′ and reverse: 5′-TCCACCACCCTGTTGCTGTA-3′ generating a 452-bp product. PCR products were analyzed on a 1% agarose gel and visualized by ethidium bromide staining. Glyceraldehyde-3-phosphate dehydrogenase (GPDH) was used as PCR amplification control [25].

RETRACTED

#### Endothelial NOS (eNOS) Immunolocalization

Since eNOS participates to CST-induced signaling and cardioprotection [9], [10], [13], [36], we tested whether CST may affect eNOS activation in post-ischemic hypertrophic hearts. Additional rat hearts (SHR_Sham: n = 3; SHR_I/R n = 3; SHR_CST-Post n = 3) were flushed in PBS, fixed in methanol: acetone: water solution (2∶2∶1), dehydrated in graded ethanol (90%–100%), cleared in xylol, embedded in paraplast (Sigma-Aldrich), and serially sectioned at 8 µm. Sections were placed onto Superfrost Plus slides (Menzel-Glaser, Braunschwerg-Germany), deparaffined in xylene, and rehydrated in an alcohol gradient [37].

For immunodetection, sections were rinsed in TBS, incubated with 1.5% BSA in TBS for 1-h, and incubated overnight at 4°C with rabbit polyclonal antibody (1∶100) directed against phospho-eNOS (1∶100; Santa Cruz Biotechnology). Signal was detected on slides washed in TBS (3×10-min), and incubated with FITC-conjugated anti-rabbit IgG (1∶100; Sigma-Aldrich). Nuclei were counterstained with Hoechst (1∶10.000; Sigma-Aldrich) for 5 min. Slides were observed using a deconvolution microscope (DMI 4000 LEICA, Wetzlar-Germany) [37].

Hearts perfused with Krebs solution alone for 190 min (Sham Group) were used to evaluate the basal level and stability of studied enzyme throughout the experiment.

### Assessment at 20 min reperfusion

#### WB for RISK pathway

Since *RISK pathway* is involved in the CST induced signaling and cardioprotection in normotensive hearts [16], we tested whether in hypertrophic hearts CST may affect *RISK pathway* activation. Samples collected immediately after the 20-min reperfusion were used in order to directly study whether CST-Post is able to induce phosphorylation of Akt, GSK3β, ERK1/2 and PKCε in early reperfusion. After stabilization (40-min), rat hearts underwent 30-min global ischemia followed by 20-min reperfusion (with and without CST). Hearts perfused with KHS alone for 90-min (Sham-short Groups) were used to evaluate the basal level and stability of phosphorylation of kinases throughout the experiment. In brief, the supernatants (60 µg proteins) [38] were subjected to SDS-PAGE on various percent of acrylamide gels (8% for PKCε, phospho-PKCε; 10% for Akt, phospho-Akt; GSK3β, phospho-GSK3β) and transferred to PVDF membranes (GE Healthcare, Buckinghamshire-UK). After blocking with non-fat dried milk (Santa Cruz Biotechnology) membranes were then incubated overnight at 4°C with the following primary antibodies: anti-Akt, anti-phospho-(Ser473)-Akt, anti-GSK3β, (Cell Signaling Technology, Beverly, MA-USA), anti-phospho-(Ser-9)-GSK3β, anti-PKCε, anti-phospho-(Ser729)-PKCε, (Santa Cruz Biotechnology). To confirm equal protein loading, membranes were incubated with an anti-β-actin antibody (Sigma-Aldrich). Immunoblotted proteins were visualized using an Immuno-Star HRP Substrate Kit (Bio-Rad Laboratories, Hercules, CA-USA) and quantified by Kodak Image Station 440CF. Image analyses were performed by Kodak 1D 3.5 software [27], [28]. Individual values (total and phosphorylated kinases) were compared to β-actin and used to calculate the phospho/total ratio of kinases. The mean value of the Sham group was considered as the reference for all groups, including Sham.

RETRACTED

#### Detection of SNO by Biotin switch assay (BS) and WB

SNO of L-type calcium channels has been implicated in cardioprotection [18], [39]. Thus, we studied whether CST may favor SNO of these channels in SHR and WKY hearts. To this purpose BS assay was performed as described [13] on ventricular homogenates collected during early reperfusion. Biotinylated samples were separated on 10% SDS-PAGE gels, transferred to membrane, blocked with non-fat dried milk and incubated with streptavidin-peroxidase (Sigma-Aldrich) diluted 1∶5000 for 1 h. The membranes used for S-nitrosylation were stripped and re-probed by using a polyclonal rabbit anti-L-type calcium channel antibody (Santa Cruz Biotechnology). Immunodetection for both WB and BS assay was performed with an enhanced chemiluminescence kit (ECL-PLUS, GE-Healthcare, Buckinghamshire-UK). Autoradiographs, obtained by exposure to X-ray films (Hyperfilm ECL, GE-Healthcare), were digitalized and the densitometric analysis of the bands was carried out using NIH IMAGE 1.6 for a Macintosh computer based on 256 grey values (0 = white; 256 = black) [13]. Individual values (total and nytrosylated channel) were compared to β-actin and used to calculate the nytrosylated/total ratio of protein channel. The mean value of the Sham group was considered as the reference for all groups, including Sham.

### Drugs

Human CST was synthesized by the solid-phase method, using 9-fluorenylmethoxy-carbonyl protection chemistry [40]. Peptide was purified to >95% homogeneity by preparative reverse-phase HPLC on C-18 silica column. Authenticity and purity of peptide was further verified by analytical chromatography (reverse-phase HPLC) and electrospray-ionization or matrix-assisted laser desorption mass spectrometry [40]. CHE, and WN were purchased from Sigma-Aldrich.

### Statistical analysis

All data are expressed as means±SEM. ANOVA followed by Bonferroni’s Multiple comparison test and Newman–Keuls multiple comparison test for post-ANOVA comparisons have been used when appropriate. Two way ANOVA was used when comparing WKY and SHR groups (Graphpad-Prism). A p value<0.05 was considered statistically significant.

## Results

### CST-Post Limits I/R Injury (infarct size and apoptosis) after 30-min ischemia and 120-min reperfusion

In order to assess the effectiveness of CST-Post in limiting I/R injury, infarct size and apoptotic indices were evaluated (***Figs 2*** and ***3***).

**Figure 3:** Apoptotic factors after 30-min ischemia and 120-min reperfusion. Representative Western Blots and relative densitometry for ARC (panel A) and for cleaved caspase 3 (panel B). Individual values were compared to β-actin and the mean value of the Sham group was considered as the reference for all groups, including Sham. Immunohistochemical localization of the apoptosis repressor recruitment domain (ARC, white arrows) in the ventricular cardiomyocytes of SHR Sham (D), SHR_I/R (E), SHR_CST-post (F) rat. Immunohistochemical localization of caspase 3 (blue arrows) of WKY (G), SHR_Sham (H), SHR_I/R (I), SHR_CST-post (L) in the ventricular cells. (C) Negative control. *p<0.01. ANOVA followed by Bonferroni’s Multiple comparison Test, (n = 6 for each group).

Infarct size (IS) is expressed as a percentage of risk area (Fig. 2, panels A and B). We confirmed that CST was able to reduce IS in WKY hearts and that, in the I/R group of SHR hearts, the IS was larger (70±11% of risk area) as compared to WKY group (Fig. 2, panel A). We found significant reduction of IS (reduced to 24±2%) in SHR_CST-Post (p<0.01 *vs.* SHR_I/R) (Fig. 2, panels A and B).

RETRACTED

The co-infusion with WN, an inhibitor of PI3K/Akt or CHE, an inhibitor of PKC, blocked the protective effects of CST-Post in SHR (IS was 54±2% and 62±2% respectively, p<0.05 *vs.* SHR_CST-Post, and p = NS (not significant) *vs.* SHR_I/R for both) (Fig. 2, panel B); similar results were observed for normal hearts [16].

CST protective effects on I/R injury were confirmed by assessing TUNEL-positive apoptotic cardiomyocytes. The apoptotic index was similar in WKY and SHR_Sham, while I/R increased the number of apoptotic cardiomyocytes in SHR_I/R (p<0.05 *vs*. SHR_Sham). CST-Post was found to significantly (p<0.05 *vs*. SHR_I/R) reduce the number of post-ischemic apoptotic myocytes (Fig. 3, panel C). Apoptotic nuclei appear to be condensed, fragmented and with dark stained nuclei (Fig. 2, panels D–G). Cardiomyocytes were discriminated from other non-myocyte cells by comparison with connexin 43 localization in parallel ventricular sections (panels I–M).

Usually, it is recommended to employ two or more distinct assays to confirm that cell death is occurring via apoptosis. Therefore, to strength data on apoptosis we performed immunoblotting analysis (Fig. 3, panels A and B) and immunohistochemical analysis (Fig. 3, panels D–L) of apoptosis repressor ARC and cleaved caspase 3. We found a significant increase of ARC (panel A) and a significant reduction of cleaved caspase 3 (panel B) in SHR_CST-Post. ARC (panels D–F) and Caspase 3 (panels G–L) immunohistochemical data confirmed immunoblotting densitometry.

In immunohistochemical analysis, labeling specificity was confirmed by the absence of the signal in parallel control sections without the primary antibody (Fig. 3, panel C).

### CST-Post improves post-ioschemic cardiac function recovery

The data of I/R injury were corroborated by post-ischemic cardiac function recovery (Table 1). CST limited the post-ischemic myocardial contracture (EDVP) in both WKY and SHR strain. Moreover CST improved post-ischemic contractile activity (dLVP) and maximal LV contraction rate (dP/dt_max_) in both strains.

**Table 1:** Pre and post ischemic cardiac function.

	WKY		SHR			
	Baseline*(Pre-isch)*	I/R*(End rep)*	CST-Post*(End rep)*	Baseline*(Pre-isch)*	I/R*(End rep)*	CST-Post*(End rep)*
**dLVP ** ***(mmHg)***	85±4	43±6**	84±16	106±4	57±12**	135±28
**+(LVdP/dt)_max_** ***(mmHg/sec)***	2713±132	1748±103**	2857±415	3290±109	2321±178*	3921±718
**EDVP ** ***(mmHg)***	5±1	35±11**	4±2	6±1	59±7**	6±1

dLVP = developed left ventricular pressure (index of contractile activity); +(LVdP/dT)max = maximal value of the first LVP derivative (index of maximal LV contraction rate); EDVP = end diastolic ventricular pressure (index of post-ischemic contracture); Pre-isch = before ischemia; End rep = at the end of reperfusion. Baseline value are the pooled data of I/R and CST-Post groups. *p<0.05 *vs.* Baseline; **p<0.005 *vs.* Baseline.

RETRACTED

At the concentration used to dissolve WN, DMSO has not effect on both I/R injury and post-ischemic cardiac function [28], [41], [42].

### CST-Post enhances eNOS and HIF-α expression

To test whether CST-Post promotes early pro-angiogenic factors, namely HIF-1α and eNOS we exposed rat ventricular sections to phospho-eNOS and HIF-1α antibodies.

In SHR_Sham (Fig. 4, panels B, C) and SHR_I/R (Fig. 4, panels D, E) the phospho-eNOS signal was localized at the level of the ventricular endocardial-endothelium and to a lesser extent on the vascular endothelium and on the myocardiocytes. After CST-Post (Fig. 4, panels F, G) phospho-eNOS expression was strongly increased in both coronary vessels and myocardiocytes.

**Figure 4:** Phospho-eNOS localization after 30-min ischemia and 120-min reperfusion. Immunolocalization of phospho-eNOS (B–G), in SHR_Sham (B, C), SHR_I/R (D, E), SHR_CST-post (F, G) rat ventricular sections. The enzyme is localized mainly in vascular (yellow arrows) and endocardial endothelium (red arrows). Negative control is shown in A. Nuclei are counterstained with Hoechst, (n = 3 for each group).

Data on expression of HIF-1α were analyzed with RT-PCR and Western Blotting analyses (Fig. 5, panels A and B). The levels of HIF-1α mRNA and protein were significantly higher in I/R group with respect to Sham. CST-Post leads to a further increase in the expression of HIF-1α protein (panel B). Immunohistochemical analyses revealed the presence of HIF-1α in ventricular cardiomyocytes. Augmented expression of HIF-1α was seen particularly in coronary vessel endothelium in I/R (panel E) as compared to Sham groups (panel D). CST-Post treatment, HIF-1α expression was found to have increased further in both cardiomyocytes and coronaries (panel F).

**Figure 5:** HIF-α expression after 30-min ischemia and 120-min reperfusion. Representative RT-PCR (panel A) and Western Blots (panel B) and relative densitometry for hypoxia-inducible factor-1α (HIF-1α). Individual values were compared to loading control and the mean value of the Sham group was considered as the reference for all groups, including Sham. Immunohistochemical localization of HIF-1α in the ventricular sections of SHR_Sham (D), SHR_I/R (E), SHR_CST-Post (F) rat. In E the inset shows a detail of HIF-1α labeled myocardiocytes. (C) Negative control. Blue arrows (cardiomyocytes), red arrows (vascular endothelium). *p<0.01. ANOVA followed by Bonferroni’s Multiple comparison test, (n = 6 for each group).

RETRACTED

Similar results were obtained in parallel experiments performed on WKY_I/R and WKY_CST-Post groups (data not shown).

In both immunofluorescence and immunohistochemical analyses, labeling specificity was confirmed by the absence of the signal in parallel control sections without the primary antibody (Figs 4A, 5C).

### CST triggers RISK pathway and SNO of calcium channel in SHR hearts after 30-min ischemia and 20-min reperfusion (Figs 6 and 7)

In order to evaluate posttranslational protein modifications induced by CST-Post, we analyzed the phosphorylation of critical proteins of the RISK pathway (Fig. 6) and the S-nitrosylation of an important component of calcium handling (Fig. 7). The representative bands and densitometric analysis of the scanned blots detected at the 20^th^-min of reperfusion in SHR hearts are presented in Fig. 6. Data are normalized with respect to the mean value of single value loading of β-actin. The infusion of CST-Post enhanced phosphorylation of all kinases analyzed. In particular, it induced a marked activation/phosphorilation of Erk1/2, PKCε and Akt with respect to I/R group. In addition, CST infusion caused increased phosphorylation/inhibition of GSK3β, which represents the putative end-effector of RISK pathway. Similar results were obtained in parallel experiments performed on WKY_I/R and WKY_CST-Post groups (data not shown).

**Figure 6:** RISK pathway activation after 30 min ischemia and 20 min reperfusion. Western blot analysis for RISK pathway at 20-min of reperfusion. Representative Western blots and relative densitometry showing that CST-Post given in early reperfusion results in an increased phosphorylation of Akt, ERK1/2, PKCε and GSK3β with respect to I/R or Sham Group. Individual values were compared to β-actin and the mean value of the Sham group was considered as the reference for all groups, including Sham. **p<0.01 *vs.* I/R_short, #p<0.05 *vs.* Sham_short. ANOVA followed by Newman–Keuls multiple comparison test, (n = 6 for each group).

**Figure 7:** S-nitrosylation of calcium channels after 30 min ischemia and 20 min reperfusion. Western blot analysis of S-nitrosylated proteins in homogenized cardiac ventricles. S-nitrosylation of membrane protein fraction and stripped membrane incubated with an anti L-type calcium channel antibody showing S-nitrosylation at the migration position corresponding to the L-type calcium channel in WKY (panel A) and SHR (panel B) hearts. Individual values were compared to β-actin and the mean value of the Sham group was considered as the reference for all groups, including Sham. *p<0.05 ANOVA followed by Newman–Keuls multiple comparison test, (n = 6 for each group).

RETRACTED

#### L-type calcium channel S-nitrosylation (Fig7)

While I/R induced a significant decrease of S-nitrosylation of L-type calcium channels in SHR strain, CST-Post increased the S-nitrosylation of calcium channels in both WKY and SHR hearts as determined by Biotin switch method in combination with Western blot (Fig. 7, panels A and B).

## Discussion

The present study indicates that CST when given in the early reperfusion in the hypertrophic heart of SHR *1)* reduces infarct size, *2)* limits apoptosis, and *3)* increases the expression of pro-angiogenetic factors, namely HIF-1α and eNOS, already two-hours after the beginning of perfusion. These effects are accompanied by the activation of the RISK pathway and calcium channel S-nitrosylation. Taken together, these results in CST-Post group strongly support a cardioprotective/proangiogenetic role of the peptide.

Several studies revealed that the effectiveness of cardioprotective protocols (*e.g.,* ischemic preconditioning and postconditioning) is blunted in the presence of *comorbidities*, such as diabetes, hypercholesterolemia, hyperglycemia, obesity or hypertension [1], [5], [6]. As shown in different models of cardiac hypertrophy, this higher ischemic susceptibility is attributed to altered levels of kinases phosphorylation [43]–[45] and an increased cell loss by apoptosis and necrosis [46]. Consistent with this point, we recently demonstrated a reduced I-PostC protection against infarct development in hypertrophic SHR hearts [5]. Accordingly, greater attention has been paid to understand the mechanisms underlying the protection of the diseased heart.

Here we report for the first time that in the SHR model the CST treatment immediately after ischemia, namely P-PostC, induced the same cardioprotective profile as ischemic pre- and post-conditioning in normotensive animals, *i.e.* CST activated PI3K/Akt, PKCε and ERK1/2, which may converge on GSK-3β, a substrate of multiple pro-survival protein kinases. Indeed, GSK-3β phosphorylation/inactivation is considered a point of convergence for multiple protective signaling pathways [15], [16], [47]. Our findings that inhibitors of PI3K/Akt and PKC blunt the CST-Post protection suggest that, also in SHR, the infarct-limiting effect of CST-Post is mechanistically linked to RISK-dependent activation. It is likely that CST reaches the threshold for eliciting cardioprotection with pharmacological PostC in SHR. Moreover, this is also the first report that CST-induced SNO of calcium channels is observed in post-ischemic phase. Of note, this posttranslational modification of a L-type calcium channel subunit has already been described in preconditioning cardioprotection by Murphy *et al.* [18], [39] and in non-ischemic hearts treated with CST by Angelone *et al.* [13]. CST-induced NOS activation [8], [9] and bioactive NO-dependent S-nitrosylation [13] are important effectors of the peptide cardio-activity. The CST-Post-elicited S-nitrosylation of L-type calcium channel may be functionally important. Notably CST can reverse the S-nitrosylation downregulation induced by I/R in SHR. The striking improvement of post-ischemic cardiac function induced by CST-Post (Table 1) might be correlated with calcium channel S-nitrosylation. In fact, due to calcium overload post-ischemic heart develops an intense contracture which compromise contractile function. The S-nitrosylation of L-type calcium channel may limit calcium overload and may allow a better functional recovery of surviving cardiomyocytes [18], [39]. This aspect deserves future studies.

RETRACTED

Since acute post-ischemic *apoptosis* followed by *maladaptive remodeling* are particularly evident in hypertrophic hearts, such as SHR heart [31], attempts have been made to develop therapeutic strategies to protect the heart against early I/R damages by reducing the onset of apoptosis and subsequent maladaptive remodeling. Therefore, we analyzed whether in SHR hearts CST-dependent protection positively modulated post-infarction cardiac repair by limiting apoptosis and triggering adaptive processes. We found that the early infusion of CST in SHR post-ischemic hearts significantly reduced apoptosis (less TUNEL-positive nuclei and cleaved caspase), concomitant with an increased ARC-expression. Remarkably, ARC is a master regulator of cell death, by inhibiting apoptosis mediated by both the death-receptor and mitochondrial pathways [31]. In the SHR model, ARC is significantly lower in cardiac tissue (our study), as well as in skeletal, and smooth muscle [31], whereas in the heart of normal animals ARC over-expression inhibits caspase-8 activation by blocking the formation of death-inducing signaling complex [33], [48].

In the context of the hypoxic stress scenario, it is of interest that we found significantly increased levels of *pro-angiogenetic* HIF-1α in SHR exposed to CST-Post with respect to I/R Group. It is known that in normal hearts HIF-1α is a key mediator of ischemic pre- and post-conditioning and its increase is detected in post-ischemic hearts few hours after the induction of the cardioprotective strategies [23], [49]. It crucially contributes to cell survival during hypoxic stress, as that occurring during ischemia [22], [23], [49]. This effect is obtained *via* activation of several critical genes [31], including NOS [36]. Consistent with this HIF-1α/eNOS interaction, we found in CST-treated SHR hearts a parallel increase in HIF-1α and eNOS expression. Therefore, it is conceivable that the induction of a CST-dependent rapid stabilization of HIF-1α under post-ischemic conditions could contribute to extend the temporal range of the cardioprotective influence of this peptide.

RETRACTED

### Translational implications

Recent evidence indicates that in both the normal and SHR hearts the full-length CgA is present and proteolytically processed to several derived peptides, such as the cardioactive and cardioprotective VS-1 [50] and CST [12]. Although the spatio-temporal aspects of the CgA intracardiac processing remain to be studied in depth, it is possible that, like VS-1, also CST can orchestrate its cardio-activity in an autocrine and paracrine manner. Current myocardial preservation strategies may be inadequate at protecting the myocardium from the acute I/R injury which occurs either on post-acute myocardial infarct (AMI) or on aortic cross-clamping and -declamping during on-pump coronary artery bypass graft surgery, especially in the presence of comorbidities [1]. Therefore, novel therapeutic strategies, such as P-PostC, are required to protect the heart against I/R injury and reduce the extent of damage in high-risk patients undergoing post-AMI reperfusion procedures or aortic cross-declamping, to preserve ventricular systolic function and improve clinical outcomes. It is possible that the lack of CST in hypertensive conditions may be responsible of the exacerbation of I/R injury. We suggest, that an early pharmacological regime with CST (*i.e.* CST-Post) may be necessary to limit reperfusion injury, especially in conditions in which the peptide is lacking.

*In conclusion,* we show that CST, given in the early reperfusion, reduces infarct size and improves cardiac function in the post-ischemic SHR hearts, activates the RISK-pathway, elicits calcium channel S-nitrosylation in early reperfusion, while increasing two-hours after the beginning of reperfusion the expression of anti-apoptotic and pro-angiogenic factors, i.e. ARC, HIF-1α and eNOS. Taken together, the data support CST as a potential modulator in the post-ischemic scenario and a therapeutic agent for protecting the heart against I/R injury despite the presence of comorbidities such as hypertension and cardiac hypertrophy.
